The article "The Functionalities and Clinical Significance of Tumor-Infiltrating Immune Cells in Esophageal Squamous Cell Carcinoma" was retracted in 2024. Reasons: signs of a paper mill; suspected computer-generated content; unreliable results or conclusions; concerns about the data.

# The Functionalities and Clinical Significance of Tumor-Infiltrating Immune Cells in Esophageal Squamous Cell Carcinoma

**DOI:** 10.1155/2021/8635381

**Published:** 2021-09-27

**Authors:** Jishuai Zhang, Haifeng Wang, Haitao Wu, Guangliang Qiang

**Affiliations:** ^1^Department of Thoracic Surgery, Feicheng Hospital Affiliated to Shandong First Medical University, Shandong Province, China; ^2^Department of Thoracic Surgery, No.1 People's Hospital of Ningyang County, Shandong Province, China; ^3^Oncology Department, No.1 People's Hospital of Ningyang County, Shandong Province, China; ^4^Department of Thoracic Surgery, China-Japan Friendship Hospital, Chaoyang District, Beijing, China

## Abstract

Tumor-infiltrating immune cells have been implicated in the tumorigenesis and progression of esophageal squamous cell carcinoma (ESCC). However, the functionalities and clinical significance of immune cells remain largely unveiled. In this study, the gene expression data from the Cancer Genome Atlas (TCGA) and Gene Expression Omnibus (GEO) were extracted. The relative infiltrating levels were estimated by single-sample gene set enrichment analysis. Some cytotoxic immune cells were attenuated, and resting cytotoxic immune cells were accumulated in ESCC. Remarkably, we also observed that infiltrating levels of macrophage M2 and resting natural killer (NK) cells were increased in nonresponders of CRT, and T cells that had anticancer activities such as activated memory CD4 and T helper 2 (Th2) cells were significantly reduced in ESCC tissues of the nonresponders. Moreover, the high infiltrations of the resting natural killer (NK) and dendritic cell (DC) were observed to result in a shorter overall survival in ESCC. Consistently, high expression of immune checkpoint genes, CTLA4 and HAVCR2, was associated with poor prognosis. Furthermore, STAT5B, a key transcription factor, as well as its target genes, involved in the regulation of T cells, was significantly downregulated in ESCC, especially subgroup I, indicating that downregulation of STAT5B might be associated with reduced T cell-mediated anticancer activity. In conclusion, the present study significantly improved our understanding of the regulatory roles of immune cells in ESCC.

## 1. Introduction

Esophageal squamous cell carcinoma (ESCC) is a major type of tumors occurring in the esophagus, accounting for more than 70% of total esophageal cancer cases worldwide [1]. The 5-year survival rate of esophageal cancer is less than 25%, which makes it one of the leading causes of cancer-related deaths [2]. Risk factors for ESCC include alcohol consumption, tobacco smoking, and other unhealthy lifestyles [3], and though the incidence of ESCC has been declining in Western countries, it still remains an important public health concern in East Asia and Africa [1].

The article "The Functionalities and Clinical Significance of Tumor-Infiltrating Immune Cells in Esophageal Squamous Cell Carcinoma" was retracted in 2024. Reasons: signs of a paper mill; suspected computer-generated content; unreliable results or conclusions; concerns about the data.

For cancers that are closely associated with chronic inflammation, such as colorectal carcinoma, hepatocellular carcinoma, and ESCC, inflammatory mediators released by immune cells are often responsible for abnormal cell proliferation, genomic instability, oncogene activation, and angiogenesis [4]. Also, responses to therapy are affected by inflammation and immunity [5]. Since immunotherapy has emerged as a promising treatment for patients with advanced-stage ESCC, many recent studies are placing emphasis on the composition and function of immune cells in tumor microenvironment, and the relationship between immune cell infiltrating and ESCC survival has attracted much attention. In a previous research, immunohistochemistry was applied to measure the infiltration of T cells and the expression of immune checkpoint proteins in ESCC patients, including PD-1, TIGIT, PD-L1, and PD-L2, and the abundance of these checkpoint proteins was found to be associated with patients' prognoses [6]. Another study has hinted that intraepithelial CD4+ lymphocyte infiltration could contribute to favorable prognosis in ESCC [7]. Moreover, the abundance of CD103 + CD8+ tumor-infiltrating lymphocytes (TILs), which was a subpopulation of CD8+ TILs, was found to be associated with better overall survival of ESCC patients [8]. Infiltration of macrophages, such as CD68+ and CD204+, in ESCC was also evaluated, and a higher CD8+/CD204+ ratio could serve as a positive prognostic indicator for ESCC patients [9].

Considering the diversity of distinct tumor-infiltrating immune cells, the landscape of immune cell infiltrating in ESCC still remains largely unveiled. Here, we estimated the relative infiltrating levels of the immune cells in ESCC and characterized their functionalities and clinical significance.

## 2. Materials and Methods

### 2.1. Data Collection

The gene expression data from the Cancer Genome Atlas (TCGA) project [10] were collected from UCSC Xena database [11]. We only retained 81 esophageal squamous cell carcinoma (ESCC) and 11 adjacent normal tissues with detailed clinical information. The expression values were normalized to log2 (FPKM (Fragment Per Kilobase Per Million Reads) +1) [12]. The gene expression data of responders and nonresponders of preoperative chemoradiotherapy (CRT) were collected from Gene Expression Omnibus (GEO) with accession GSE45670 and normalized by MAS5 (MicroArray Suite 5.0) by previous study [13].

### 2.2. Estimation of Infiltrating Levels

A total of 570 genes representing 26 types of immune cells, fibroblast, and endothelial cells were collected from previous study. The relative infiltrating levels were estimated by single-sample gene set enrichment analysis (ssGSEA), which were implemented in R *gsva* package [14]. Single-sample GSEA (ssGSEA), an extension of Gene Set Enrichment Analysis (GSEA), calculates separate enrichment scores for each pairing of a sample and gene set. Each ssGSEA enrichment score represents the degree to which the genes in a particular gene set are coordinately up- or downregulated within a sample.

The article "The Functionalities and Clinical Significance of Tumor-Infiltrating Immune Cells in Esophageal Squamous Cell Carcinoma" was retracted in 2024. Reasons: signs of a paper mill; suspected computer-generated content; unreliable results or conclusions; concerns about the data.

### 2.3. Overrepresentation Enrichment Analysis

Prior to the overrepresentation enrichment analysis, we identified the differentially expressed genes in each subgroup by pairwise Wilcoxon rank-sum test and fold change methods (FDR < 0.05 and fold change > 2) [15]. The overrepresentation enrichment analysis was implemented in R *clusterProfiler* package [16, 17].

### 2.4. Hierarchical Clustering Analysis

The gastric cancer samples were clustered based on the infiltrating levels of the 28 cells. The Ward method and Euclidean distance were used in this analysis. The default options were selected for the other parameters.

### 2.5. Survival Analysis

The univariable Cox proportional hazard regression analysis was used to identify infiltrating cells associated with overall survival. The survival analysis was implemented in R *survival* and visualized by R survminer package.

## 3. Results

### 3.1. The Differential Infiltrating Cells between Esophageal Squamous Cell Carcinoma and Adjacent Normal Tissues

In this study, we collected gene expression data of 81 esophageal squamous cell carcinoma (ESCC) and 11 adjacent normal tissues from the Cancer Genomics Atlas (TCGA). The relative infiltrating levels of 28 cells in ESCC and adjacent normal tissues were estimated by the single-sample enrichment analysis (ssGSEA). Among these cells, 11 were differentially infiltrated into ESCC tissues, of which, endothelial cells and resting CD4 memory cells were found to be decreased in ESCC (Figure 1(a)). Particularly, macrophage M1, regulatory T cells (Tregs), and T helper 1 cells (Th1) were significantly infiltrated into ESCC tissues, and their corresponding marker genes were observed highly expressed in ESCC (Figure 1(b)). These results indicated that the immune cells were highly coinfiltrated into the ESCC tissues, and the ESCC tissues exhibited an inflammatory phenotype.

### 3.2. The Association between Tumor-Infiltrating Immune Cells and Response of Preoperative Chemoradiotherapy (CRT)

As the immune cells were associated with the response of drug treatment, we collected the gene expression data of responders and nonresponders of preoperative CRT. The differential analysis revealed that infiltrating levels of macrophage M2 and resting natural killer (NK) cells were increased in nonresponder ESCC tissues (Figures 2(a) and 2(b), Wilcoxon rank-sum test, *P* < 0.05), suggesting that macrophage M2 and resting NK cells might be associated with the resistance of CRT. In contrast, the T cells that had anticancer activities such as activated memory CD4 and T helper 2 (Th2) cells were significantly reduced in ESCC tissues of the nonresponders, suggesting that these cells mediated anticancer activity might promote the sensitivity of CRT in ESCC. These results revealed that the tumor-infiltrating levels of immune cells were closely associated with the response of CRT in ESCC.

The article "The Functionalities and Clinical Significance of Tumor-Infiltrating Immune Cells in Esophageal Squamous Cell Carcinoma" was retracted in 2024. Reasons: signs of a paper mill; suspected computer-generated content; unreliable results or conclusions; concerns about the data.

### 3.3. Immune Subtypes of ESCC Samples

As the ESCC samples exhibited variable infiltrating levels of immune cells due to intertumor heterogeneity, we classified the ESCC samples into three subgroups based on the infiltrating levels of immune cells by hierarchical clustering analysis. As shown in Figure 3(a), the subgroups II and III had significantly higher immune cell infiltrating levels than subgroup I. The survival analysis revealed that subgroup I had a better prognosis than the other two subgroups (Figure 3(b)), suggesting that the high infiltration of immune cells might be associated with poor prognosis. Particularly, high infiltrations of the resting natural killer (NK) and dendritic cell (DC) were observed to result in a shorter overall survival in ESCC (Figures 3(c) and 3(d)). These results indicated that the immune profiles were significantly different and associated with overall survival in ESCC samples.

### 3.4. The Immune Checkpoints in ESCC

As the inflammatory phenotypes were observed in ESCC, we attempted to examine whether the immune checkpoints were associated with the immune evasion in ESCC. Based on the three immune subgroups in ESCC, we found that CTLA4 and HAVCR2 (TIM-3) were significantly upregulated in subgroups II and III (Figures 4(a) and 4(b)). CTLA4 and TIM-3 were well-known regulators of inhibiting the anticancer activity of immune cells. These results indicated that the immune checkpoint inhibitors might be applied to the treatment of ESCC samples with higher infiltration of immune cells.

### 3.5. The Downregulated Genes and Pathways in ESCC

As the upregulated signatures were characterized by the inflammatory phenotypes in ESCC, we then investigated the downregulated genes and pathways. We found that the synthesis and metabolic activity-related pathways were significantly attenuated in ESCC (Figure 5(a)). Furthermore, we also found the STAT5B, a key transcription factor involved in the regulation of T cells, was significantly downregulated in ESCC, especially subgroup I (Figure 5(b)). Consistently, the lower expressions were observed in target genes of STAT5B such as ENPP2, TAL1, CD247, SLAMF1, IRF4, BATF, and IRF8. These results indicated that downregulation of STAT5B might be associated with reduced T cell-mediated anticancer activity.

The article "The Functionalities and Clinical Significance of Tumor-Infiltrating Immune Cells in Esophageal Squamous Cell Carcinoma" was retracted in 2024. Reasons: signs of a paper mill; suspected computer-generated content; unreliable results or conclusions; concerns about the data.

## 4. Discussion

Tumor-infiltrating immune cells play a role in the regulation of tumor progression and are often found in esophageal squamous cell carcinoma (ESCC). However, the landscape of immune cell infiltrating in ESCC still remains largely unveiled. In this study, we estimated the infiltrating levels of immune cells in 81 ESCC and 11 adjacent normal tissues. Macrophage M1, regulatory T cells (Tregs), and T helper 1 cells (Th1) were significantly infiltrated into ESCC tissues, and their corresponding marker genes were observed highly expressed in ESCC (Figure 1(b)). Particularly, Tregs and Th1 were dysregulated and contributed to the initiation and propagation in ESCC [18]. The high infiltration of these cells showed that the functionalities of these immune cells might be impaired in ESCC. As the immune cells were associated with the response of drug treatment [19], we observed that infiltrating levels of macrophage M2 and resting natural killer (NK) cells were increased in nonresponders of CRT, and T cells that had anticancer activities such as activated memory CD4 and T helper 2 (Th2) cells were significantly reduced in ESCC tissues of the nonresponders. In accordance with these results, M2 has been found to result in poor response of chemotherapy [20], and increased infiltration of activated memory CD4 in ESCC patients with chemoradiotherapy was a favorable indicator of ESCC prognosis [21].

As the ESCC samples exhibited variable infiltrating levels of immune cells due to intertumor heterogeneity, we found that the ESCC samples could be classified into three subgroups based on the infiltrating levels of immune cells. The worse prognosis in patients with high infiltration of immune cells was also observed by previous study [22]. Particularly, high infiltrations of the resting natural killer (NK) and dendritic cell (DC) were observed to result in a shorter overall survival in ESCC (Figures 3(c) and 3(d)). The attenuated cytotoxicity in NK and DC might be the cause of poor prognosis. Notably, CTLA4 and HAVCR2 (TIM-3) were significantly upregulated in subgroups II and III (Figures 4(a) and 4(b)). High expression of CTLA4 and HAVCR2 was associated with poor prognosis [23, 24], and the two proteins might be the potential immunotherapeutic targets in ESCC [25].

As the upregulated signatures were characterized by the inflammatory phenotypes in ESCC, we found that the synthesis and metabolic activity-related pathways were significantly attenuated in ESCC, suggesting that the normal function of esophagus might be impaired [26, 27]. Furthermore, we also found the STAT5B, a key transcription factor involved in the regulation of T cells, was significantly downregulated in ESCC, especially subgroup I (Figure 5(b)). Consistently, the lower expressions were observed in target genes of STAT5B such as ENPP2, TAL1, CD247, SLAMF1, IRF4, BATF, and IRF8, indicating that downregulation of STAT5B might be associated with reduced T cell-mediated anticancer activity.

The article "The Functionalities and Clinical Significance of Tumor-Infiltrating Immune Cells in Esophageal Squamous Cell Carcinoma" was retracted in 2024. Reasons: signs of a paper mill; suspected computer-generated content; unreliable results or conclusions; concerns about the data.

There are some limitations in our study. First, it lacks the validation by our own data. Second, in vitro and in vivo experiments are still needed to validate.

In summary, the present study systematically characterized the immune cells infiltrated in the ESCC tissues and identified some key immune cells associated with CRT, and key regulators implicated in ESCC.

## Figures and Tables

**Figure 1:** The differentially infiltrating levels of immune cells between ESCC and adjacent normal tissues. (a) The differentially infiltrating immune cells and their infiltrating levels in ESCC and normal tissues. (b) The expression patterns of marker genes in macrophage M1, Tregs, and Th1. The expression levels were scaled at -3 to 3. ^∗∗∗∗^*P* < 0.0001.

**Figure 2:** The immune cells associated with the response of chemoradiotherapy. The infiltrating levels of macrophage M2, resting NK cells, activated memory CD4 cells, and Th2 are displayed in (a–d). ^∗^*P* < 0.05.

**Figure 3:** The immune subtypes and clinical significance in ESCC. (a) The hierarchical clustering of the ESCC samples by the infiltrating levels of immune cell. (b) The prognostic difference between subtypes I and others. (c, d) The prognostic significance of resting DC and NK cells, respectively.

**Figure 4:** The expression patterns of immune checkpoint genes in the immune subtypes. The upregulations of two immune checkpoint genes, CTLA4 and HAVCR2 (TIM-3), in subtypes II and III are displayed in (a, b), respectively. ^∗∗∗∗^*P* < 0.0001.

**Figure 5:** The aberrantly inactivated pathways in ESCC. (a) The pathways enriched by downregulated genes in ESCC. The node size represents the number of genes included in the pathway, and the node color represents the statistical significance. (b) The STAT5B expression pattern in normal tissues and immune subtypes. (c) The downregulated target genes of STAT5B. ^∗∗∗∗^*P* < 0.0001.

## Data Availability

All the data can be downloaded from the Cancer Genome Atlas (TCGA) and Gene Expression Omnibus (GEO) with accession GSE45670.
